# The Effect of MDT Collaborative Nursing Combined with Hierarchical Nursing Management Model on the Quality of Life and Comfort of Patients with Gallbladder Stones Combined with Acute Cholecystitis after Surgery

This article has been retracted.

**DOI:** 10.1155/2022/8696084

**Published:** 2022-06-13

**Authors:** Li Lu, Jun Yang, Jiafeng Zheng, Chenchen Zhang, Ye Yang, Juan Huang

**Affiliations:** ^1^Department of Hepatobiliary Surgery, Wuhan No. 1 Hospital, China; ^2^Intensive Care Unit, Wuhan Wuchang Hospital, Wuchang Hospital Affiliated to Wuhan University of Science and Technology, China

## Abstract

**Objective:**

To explore the effect of MDT (multidisciplinary team) collaborative nursing combined with hierarchical nursing management mode on the quality of life and comfort of patients with gallbladder stones combined with acute cholecystitis after surgery.

**Methods:**

A total of 120 patients with gallbladder stones and acute cholecystitis who were treated in our hospital from March 2019 to March 2021 were selected as prospective research objects. According to the order of care, they were divided into control group and observation group with 60 cases each. Among them, the control group implements a hierarchical nursing management model, and the observation group implements MDT collaborative nursing based on this and compares the impact of the two groups on patient's quality of life scores, daily self-care ability, nursing satisfaction, and comfort after nursing.

**Results:**

Before nursing, the comparison of the quality of life score, nursing comfort, and nursing ability of the two groups of patients was not statistically significant (*P* > 0.05). After nursing, the mental vitality score, social interaction score, emotional restriction score, and mental status of the observation group were significantly higher than those of the control group. Statistics showed that the difference was statistically significant (*P* < 0.05). After nursing, the scores of social comfort, physical comfort, and psychological comfort of the observation group were significantly higher than those of the control group, and statistics showed that the difference was statistically significant (*P* < 0.05). The health knowledge level, self-care skills, self-care responsibility, and self-concept of the observation group after nursing were higher than those of the control group, while the score of depression and mood disorder was significantly lower than that of the control group. Statistics showed that this difference was statistically significant (*P* < 0.05). After nursing, patients in the observation group had higher operating technique scores, service attitude scores, health education scores, psychological intervention scores, and nursing quality scores than those of the control group. Statistics showed that the difference was statistically significant (*P* < 0.05).

**Conclusion:**

MDT collaborative nursing combined with hierarchical nursing management mode can effectively improve the self-care ability of patients with gallbladder stones complicated with acute cholecystitis, effectively improve the quality of life of patients, and improve the satisfaction and comfort of patients with nursing care. The postnursing care of patients after inflammation has a certain reference value.

## 1. Introduction

Acute cholecystitis is a common complication of gallbladder stones. It usually has sudden onset and severe pain, most of which are accompanied by vomiting, nausea, and other symptoms. Laparoscopic cholecystectomy is often used to treat gallbladder stones with acute cholecystitis, and nursing interventions are taken to reduce postoperative complications and shorten the length of hospital stay, thereby improving the quality of life and nursing satisfaction [1]. Gallbladder stones with acute cholecystitis are more common in middle-aged and elderly people and are often associated with basic diseases such as lung disease, diabetes, and hypertension. They have decreased immune function, low pain tolerance, and high risk of postoperative complications, which is not conducive to postoperative recovery [2]. Taking active and effective nursing measures can improve the effect of surgery, reduce complications, and speed up the recovery process after surgery. Cholecystectomy is often used in clinical treatment. However, if you want to improve the quality of life of patients, you need to provide hierarchical care and management to patients [3]. This model mainly implements hierarchical management by setting up corresponding levels of nurses, that is, the head nurse assigns tasks and supervises the implementation, and the senior responsible nurses, junior responsible nurses, and assistant nurses carry out specific nursing work [4]. Through the use of this method, medical resources are effectively allocated, and the fatigue of nurses is effectively relieved, and at the same time, the work is carried out in an orderly manner, which greatly improves the quality of care and establishes a good doctor-patient relationship. But there are still many shortcomings [5]. MDT collaborative care is a newly emerging nursing model in recent years, which is obviously scientific and holistic, and can effectively avoid the adverse effects of the limitation of knowledge domains on patient treatment and even the formation of wrong decisions [6, 7]. In addition, gallbladder stones combined with acute cholecystitis in a very complicated individual part of patients are often involved in systemic multiorgan dysfunction. Multidisciplinary collaborative nursing can put forward more standardized, reasonable, and best nursing advice through professional integration [8]. Therefore, this study explored the effect of MDT collaborative nursing combined with hierarchical nursing management mode on the quality of life and comfort of patients with acute cholecystitis after gallbladder stone surgery and provided a reference for clinical care after surgery for gallbladder stones with acute cholecystitis.

## 2. Information and Methods

### 2.1. Research Object

A total of 120 patients with gallbladder stones and acute cholecystitis who were treated and nursed in our hospital from March 2019 to March 2021 were selected as the research objects, and they were divided into a control group and an observation group with 60 cases each. There were 60 patients in the control group, including 29 males and 31 females, with an average age of 50-78 (66.2 ± 6.14) years old and an average illness time of 3-17 years (9.1 ± 2.7) years. There were 29 cases of multiple stones and 31 cases of single stones.. There were 13 cases of junior college or above, 17 cases of junior high school, and 20 cases of elementary school and illiterate; 60 cases of observation group, 27 males and 33 females, age 49-79 average (67.4 ± 7.09) years old, sick time 4-19. In an average of 10.1 ± 1.7 years, there were 26 cases of multiple stones and 34 cases of single stones. There were 11 cases of a college degree and above, 19 cases of junior high school, and 20 cases of elementary school and illiterate. Statistics of general data of the two groups of patients, such as gender, age, and time of illness, showed that the difference was not statistically significant (*P* > 0.05).

### 2.2. Patient Eligibility Criteria

Inclusion criteria were as follows: (1) the included patients comply with the “Consensus Opinions on the Medical Diagnosis and Treatment of Chronic Cholecystitis and Gallbladder Stones” [9] according to the diagnosis basis of gallbladder stones with acute cholecystitis: acid reflux, belching, stomach burning, abdominal distension, bitter mouth, etc. Symptoms, after B-ultrasound examination, gallbladder wall thickening, gallbladder fossa effusion, and positive Murphy's sign; (2) able to strictly follow the doctor's instructions to complete the relevant treatment work, the condition is stable, without other cardiovascular diseases, and the patient and family members voluntarily participate in the treatment. (3) accompanied by obvious abdominal muscle rigidity, abdominal pain, increased white blood cell count, abdominal X-ray examination revealed free gas under the diaphragm, and abnormal serum total bilirubin in some patients. Exclusion criteria were as follows: (1) those with other immune diseases, malignant tumors, or incomplete medical records, those with autoimmune system diseases, those with mental illness, and those who cannot communicate normally; (2) those with gangrenous and purulent cholecystitis and those with abnormal hematopoietic system and abnormal cardiopulmonary function; and (3) patients with cognitive dysfunction, surgical contraindications, severe liver and kidney disease, blood system disease, etc.

### 2.3. Method

#### 2.3.1. Level Nursing Management Nursing

Among them, the control group implements a hierarchical nursing management model, that is, four personnel are arranged for each ward, namely, the head nurse, senior responsible nurse, junior responsible nurse, and assistant nurse, and the head nurse arranges corresponding work content and solves daily work problems. Senior responsible nurses arrange corresponding work content for junior responsible nurses and assistant nurses, which mainly include evaluating the basic data of patients and doing preoperative preparations, intraoperative observations, and postoperative nursing. At the same time, the primary responsible nurse and the assistant nurse also need to communicate with the patient, inform the patient of the surgical method, purpose, and postoperative precautions, so as to eliminate the patient's fear, and then cooperate with the treatment. In addition, senior responsible nurses need to formulate strict diet and medication plans for patients. Primary responsible nurses need to strictly follow the diet and medication plan to care for the patients and strengthen the observation of the patient's vital signs and adverse reactions. Once abnormalities occur, they need to be reported to the doctor for treatment in time. Assistant nurses need to cooperate with patients in daily care and at the same time take care of the daily life of patients.

#### 2.3.2. MDT Collaborative Care

Establish a nursing intervention team: set up an MDT collaborative nursing team according to the purpose of the research. The members include attending physicians, nutritionists, nursing staff, and psychological counselors, etc., to assess and evaluate their clinical knowledge and skills and to strengthen comprehensive quality training and deepen it. The concept of serving others: at the same time, scientific evaluation of the patient's condition, mental state, etc. is made on this basis, and targeted nursing intervention programs are formulated. After receiving the consultation, the nursing staff is responsible for the basic nursing work of the patient after admission, and the basic information of the patient is integrated and analyzed, including general information such as age, address, and clinical data such as drug allergy history and surgical contraindications, as the basic data of the group consultation for analysis. Nursing plan revision provides reference. The responsible nurse conducts ward rounds every day, feedbacks the patient's treatment progress to the nursing team, at the same time summarizes the difficult points in the treatment and nursing work, includes the patient into the clinical nursing path, and strengthens the observation of the patient's condition change. If there are uncomfortable symptoms such as “abdominal pain, nausea, and vomiting,” the nursing staff should promptly report to the medical staff to deal with it; the diet should be “high-calorie, high-fiber, and high-protein.” Wait for food, pay attention to the gastrointestinal preparation 1d before surgery; adjust the patient's position 6 h after surgery, go to the pillow and lie supine and assist with gentle massage, then turn over once every 2 h, and guide the patient after the patient's condition is stable Get out of bed; properly fix the drainage tube after the operation to prevent the patient from turning over and causing the tube to bend or fall off. At the same time, the nursing staff should strengthen the nursing accident record and make detailed notes, which can facilitate the summary of experience and improve the clinical nursing path table. Before the consultation, the nursing staff should analyze the evaluation data during the hospitalization in detail, and then during the consultation, the members of different disciplines can discuss and ask questions according to the specific situation of the patient and then formulate treatment and nursing plans. According to the results of MDT collaborative nursing, the patient's condition and evaluation results are summarized, and then members are organized to participate in the discussion and to put forward reasonable nursing opinions in various disciplines through brainstorming.

### 2.4. Observation Indicators

(1) Comfort: the content of comfort evaluation includes three items: social comfort, physical comfort, and psychological comfort. The maximum score for each item is 100 points. The higher the score, the better the comfort. (2) Self-care ability assessment form: includes 43 items in 4 dimensions, namely, health knowledge level (14 items), self-care skills (12 items), self-care responsibility (8 items), and self-concept (9 items). Each item has 5 points, 11 of which are reverse scores, with a full score of 172 points. The higher the score, the stronger the self-care ability. The Cronbach's *α* values measured on the above scales before use were all greater than 0.914. The patient fills in independently without being affected by any internal or external factors, and the test will be completed within 30 minutes. (3) Quality of life score: includes four parts: mental vitality score, social interaction score, emotional restriction score, and mental status score. Each part is scored from 0 to 100 points. The higher the score, the better the quality of life of patients with urinary tract infection. The quality of life score is the simplest and commonly used method to evaluate the quality of life of patients. It is easy for patients to understand and accept, and has good reliability and validity. The measured Cronbach's *α* value is greater than 0.962, and it is highly sensitive and convenient for recording. (4) Postnursing satisfaction: a satisfaction questionnaire is issued from the patient's admission. The content of the survey includes postnursing operation techniques, service attitudes, health education, psychological intervention, and nursing quality satisfaction. Each item is scored 1-10 points, the higher the score it shows, the higher the patient's satisfaction. The clinical research process is shown in Figure 1.

### 2.5. Statistical Methods

We use Epidata to enter all the data and then use SPSS 25.0 to statistically process the data. The data needs to be entered into the computer database by a second person to ensure the completeness and accuracy of the data. The measurement data was represented by mean ± standard deviation ($\bar{x}\pm \text{S}$) using the one-way variance test, and the counting data was represented by the percentage (%) using the *χ*^2^ test, which are statistically significant at *P* < 0.05.

## 3. Results

### 3.1. Comparison of Quality of Life Scores

Before nursing, the comparison of the quality of life scores of the two groups of patients was not statistically significant (*P* > 0.05). After nursing, the mental vitality score, social interaction score, emotional restriction score, and mental status of the observation group were significantly higher than those of the control group. Statistics showed that the difference was statistically significant (*P* < 0.05), see Table 1.

### 3.2. Comparison of Nursing Comfort

Before nursing, the nursing comfort of the two groups of patients was not statistically significant (*P* > 0.05). After nursing, the scores of social comfort, physical comfort, and psychological comfort of the observation group were significantly higher than those of the control group. Statistics show that this difference is statistically and academically significant (*P* < 0.05), see Table 2.

### 3.3. Nursing Ability Comparison

Before nursing, there was no significant difference in nursing ability and anxiety and depression scores between the two groups of patients (*P* > 0.05). After nursing, the observation group's health knowledge level, self-care skills, self-care responsibility, and self-concept were higher than those of the control group, while the depression mood disorder score was significantly lower than that of the control group. Statistics showed that the difference was statistically significant (*P* < 0.05), see Table 3.

### 3.4. Comparison of Nursing Satisfaction

After nursing, patients in the observation group had higher operating technique scores, service attitude scores, health education scores, psychological intervention scores, and nursing quality scores than those of the control group. Statistics showed that the difference was statistically significant (*P* < 0.05), see Table 4.

## 4. Discussion

Cholecystitis refers to the process of acute and chronic inflammation in the gallbladder caused by gallbladder stones or other reasons. It is a relatively common digestive system disease. For chronic cholecystitis, it often coexists with gallbladder stones for a long time, although the symptoms are not serious. But it often affects the quality of life of patients [10–13]. Acute calculous cholecystitis is more common in women, and its incidence is three times that of men before the age of 50. Acute acalculous cholecystitis is more common in elderly patients with severe illness and has a serious impact on the physical and mental health of patients [14, 15].

After nursing in this study, the mental vitality score, social interaction score, emotional restriction score, and mental status of the observation group were significantly higher than those of the control group, indicating that the MDT collaborative nursing combined with hierarchical nursing management model can effectively improve the patients with gallbladder stones and acute cholecystitis after surgery and self-care ability in daily life. The reasons for the analysis are as follows: MDT collaborative nursing combined with hierarchical nursing can effectively improve the active nursing awareness of nursing staff, enable them to carry out nursing work in an orderly manner, make them carry out nursing operations purposefully, and ultimately improve the quality of nursing and quality of life [16]. MDT collaborative care combined with hierarchical care is beneficial to avoid maintaining the patency of the patient's respiratory tract and reduce complications such as respiratory tract infections [13]. Wound cushion placement and ward environmental care are beneficial to reduce the pain of patients, keep the ward environment clean and tidy, increase comfort, improve their quality of life [14], and improve their satisfaction with nursing work. Drainage tube and drainage bag nursing is beneficial to maintain the patency of the drainage tube, make it fully drain, and improve the cleanliness of the drainage, effectively avoiding infection [15].

After nursing in this study, the scores of social comfort, physical comfort, and psychological comfort of the observation group were significantly higher than those of the control group. The MDT collaborative nursing combined hierarchical nursing management model can effectively improve the comfort of patients, because the MDT collaborative nursing combined hierarchical nursing management model can standardize the diet structure, improve the body's defense capabilities, and effectively establish a standardized lifestyle and eating habits, which will help improve the quality of life in the future. At the same time, with emotional nursing, it can target depression, anxiety, and other emotions of patients, carry out submissive psychotherapy, adjust the patient's emotions, and encourage them to maintain an optimistic and positive attitude [17–20]. The MDT collaborative nursing joint-level nursing management model emphasizes the “patient-centered” nursing concept, details the physical and psychological aspects of nursing, and can provide patients with high-quality, professional, and comprehensive nursing services and provide social, physical, emotional, physiological, other aspects, and social support, so as to maximize the physical and psychological comfort of patients, and improve negative emotions [21–24].

After nursing in this study, the health knowledge level, self-care skills, self-care responsibility, and self-concept of the observation group were higher than those of the control group. The MDT collaborative nursing combined hierarchical nursing management model can effectively improve the patient's nursing ability. The MDT model demonstrates that the MDT collaborative nursing joint-level nursing management model can effectively improve the self-care ability of patients through the establishment of an MDT nursing team. Multidisciplinary professionals jointly formulate and implement scientific nursing plans, which can improve the overall nursing effect and efficiency [25]. At the same time, in the perioperative period, the responsibilities of each member of the team are clarified. For example, the psychologist can relieve negative emotions such as anxiety and tension in a targeted manner and improve treatment confidence. Specialist nursing staff conduct preoperative education to improve the patient's treatment cooperation, actively communicate with the patient during the operation to relax them, and closely observe the vital signs after the operation [26, 27]. The attending surgeon minimised discomfort during the operation by being stable, precise, and light, and the dietician developed a postoperative nutritional program to aid recovery, which was enhanced by consultations.

After nursing in this study, the observation group's operating technique scores, service attitude scores, health education scores, psychological intervention scores, and nursing quality scores were higher than those of the control group. The MDT collaborative nursing combined hierarchical nursing management model can effectively improve patient satisfaction. MDT collaborative care provides patients with the best diagnosis and treatment plan, improves the diagnosis and treatment ability and academic level of the subject, promotes the true integration of medical education, research, and health management, and promotes the progress of medical science as the core goal [28–31]. MDT collaborative care is applicable to all disciplines. Through MDT collaborative care, we can fully communicate with patients and then find the most suitable scientific and reasonable comprehensive diagnosis and treatment plan for the patient's condition, so that the patient can obtain the best curative effect under the premise of ensuring medical safety [21]. The multiscientific collaboration model adjusts the mental state of patients, timely conducts health education, guides patients to take medicine, etc., ensures that patients can take in sufficient nutrition, regularly analyzes the health status of patients for treatment, can adjust plans in time, and carry out targeted care. At the same time, it is also responsible for the recovery exercise of patients' postoperative rehabilitation and self-life ability [32–35].

This research is innovative and has some limitations. The selected patients are all patients treated or cared for in our hospital, so the selection of patients to be excluded is subjective and the results of the study may be unrepresentative or biased. To sum up, the MDT collaborative nursing combined hierarchical nursing management model can effectively improve the self-care ability of patients with gallbladder stones after acute cholecystitis, effectively improve the quality of life of patients, and improve the satisfaction and comfort of patients with care. Postnursing care for patients with acute cholecystitis after surgery has a certain reference value.

## Figures and Tables

**Figure 1:** Clinical research process.

**Table 1:** Comparison of quality of life scores between the two groups ($\overset{¯}{x}\pm \text{s}$).

Group	Mental vitality score		Social interaction score		Emotional restriction score		Mental status score	
	Before care	After care	Before care	After care	Before care	After care	Before care	After care
Control group (60)	56.30 ± 9.23	89.77 ± 8.14	56.34 ± 4.25	90.25 ± 7.82	69.23 ± 10.57	95.07 ± 10.14	69.76 ± 9.15	85.45 ± 4.15
Observation group (60)	56.30 ± 9.22	97.37 ± 8.20	56.33 ± 4.24	96.27 ± 5.31	69.24 ± 10.53	99.23 ± 10.26	69.75 ± 9.26	90.03 ± 6.16
*t*	<0.001	-4.557	0.008	-4.412	-0.005	-2.008	0.005	-4.272
*P*	1.000	<0.001	0.994	<0.001	0.996	0.048	0.996	<0.001

**Table 2:** Comparison of nursing comfort between the two groups ($\overset{¯}{x}\pm \text{s}$).

Group	Social comfort score		Physiological comfort score		Psychological comfort score	
	Before care	After care	Before care	After care	Before care	After care
Control group (60)	53.40 ± 12.23	75.27 ± 6.14	54.34 ± 9.25	74.25 ± 5.82	57.31 ± 11.51	85.03 ± 2.24
Observation group (60)	52.45 ± 11.22	89.37 ± 8.20	55.33 ± 7.24	97.27 ± 2.31	59.30 ± 9.52	96.35 ± 1.26
*t*	0.443	-10.662	0.653	-28.477	-1.032	-34.118
*P*	0.658	<0.001	0.515	<0.001	0.304	<0.001

**Table 3:** Comparison of the nursing ability of the two groups of patients ($\overset{¯}{x}\pm \text{s}$).

Group	Health knowledge level		Self-care skills		Sense of responsibility	
	Before care	After care	Before care	After care	Before care	After care
Control group (60)	33.40 ± 2.23	35.27 ± 2.14	22.34 ± 6.25	24.25 ± 7.82	12.31 ± 2.51	16.03 ± 2.24
Observation group (60)	33.45 ± 2.22	38.37 ± 4.20	22.33 ± 6.24	31.27 ± 7.31	12.30 ± 2.52	23.35 ± 1.26
*t*	-0.251	-10.389	0.018	-10.369	0.044	-45.034
*P*	0.802	<0.001	0.986	<0.001	0.965	<0.001

**Table 4:** Comparison of nursing satisfaction between the two groups of patients (*x* ± s).

Group	Health education score	Psychological intervention score	Service attitude score	Operational technology score	Care quality score
Control group (60)	6.40 ± 0.18	5.27 ± 0.29	5.34 ± 0.21	5.25 ± 0.35	6.27 ± 0.14
Observation group (60)	9.45 ± 0.27	9.37 ± 0.35	9.33 ± 0.28	9.27 ± 0.33	9.39 ± 0.20
*t*	-72.805	-69.871	-88.304	-64.732	-98.994
*P*	<0.001	<0.001	<0.001	<0.001	<0.001

## Data Availability

No data were used to support this study.

## References

[1] Kimura Y., Takada T., Strasberg S. M. (2013). TG13 current terminology, etiology, and epidemiology of acute cholangitis and cholecystitis. *Journal of Hepato-Biliary-Pancreatic Sciences*.

[2] Rice C. P., Vaishnavi K. B., Chao C. (2019). Operative complications and economic outcomes of cholecystectomy for acute cholecystitis. *World Journal of Gastroenterology*.

[3] Menéndez-Sánchez P., León-Salinas C., Amo-Salas M., Méndez-Cea B., García-Carranza A. (2019). Association of laboratory and radiologic parameters in the diagnosis of acute cholecystitis. *Revista de Gastroenterología de México*.

[4] Kimura Y., Takada T., Kawarada Y. (2007). Definitions, pathophysiology, and epidemiology of acute cholangitis and cholecystitis: Tokyo guidelines. *Journal of Hepato-Biliary-Pancreatic Surgery*.

[5] Loozen C. S., Oor J. E., van Ramshorst B., van Santvoort H. C., Boerma D. (2017). Conservative treatment of acute cholecystitis: a systematic review and pooled analysis. *Surgical Endoscopy*.

[6] Battaglia A., De Meerleer G., Tosco L. (2019). Novel insights into the management of oligometastatic prostate cancer: a comprehensive review. *European urology oncology*.

[7] Garcia A. N., Costa L. D. C. M., Hancock M. J. (2018). McKenzie method of mechanical diagnosis and therapy was slightly more effective than placebo for pain, but not for disability, in patients with chronic non-specific low back pain: a randomised placebo controlled trial with short and longer term follow-up. *British Journal of Sports Medicine*.

[8] Taberna M., Gil Moncayo F., Jané-Salas E. (2020). The multidisciplinary team (MDT) approach and quality of care. *Frontiers in Oncology*.

[9] Editorial Committee of Chinese Journal of digestion (2015). Consensus opinion on medical diagnosis and treatment of chronic cholecystitis and gallbladder stones in China (2014, Shanghai). *Journal of Clinical Hepatobiliary Diseases*.

[10] Roulin D., Saadi A., Di Mare L., Demartines N., Halkic N. (2016). Early versus delayed cholecystectomy for acute cholecystitis, are the 72 hours still the rule?: a randomized trial. *Annals of Surgery*.

[11] Hirota M., Takada T., Kawarada Y. (2007). Diagnostic criteria and severity assessment of acute cholecystitis: Tokyo guidelines. *Journal of Hepato-Biliary-Pancreatic Surgery*.

[12] Karas P. L., Rankin N. M., Stone E. (2020). Medicolegal considerations in multidisciplinary cancer care. *JTO Clinical and Research Reports*.

[13] Stone E., Rankin N., Currow D., Fong K. M., Phillips J. L., Shaw T. (2020). Optimizing lung cancer MDT data for maximum clinical impact-a scoping literature review. *Translational lung cancer research*.

[14] Prabhakar C. N., Fong K. M., Peake M. D., Lam D. C., Barnes D. J. (2015). The effectiveness of lung cancer MDT and the role of respiratory physicians. *Respirology*.

[15] Tsai C. H., Hsieh H. F., Lai T. W., Kung P. T., Kuo W. Y., Tsai W. C. (2020). Effect of multidisciplinary team care on the risk of recurrence in breast cancer patients: a national matched cohort study. *Breast*.

[16] Du Z., Huang W., Wang Z. W. (2020). Application of multidisciplinary team (MDT) in the treatment of severe trauma. *Beijing Da Xue Xue Bao Yi Xue Ban*.

[17] Wennberg L., Widgren S., Axelsson R., Gerok-Andersson K., Åkerlund B. (2019). Multidisciplinary diabetic foot care in Sweden - a national survey. *Diabetes Research and Clinical Practice*.

[18] Maeng C. H., Ahn H. K., Oh S. Y., Lim S., Kim B. S., Kim D. Y. (2020). Practice patterns of multidisciplinary team meetings in Korean cancer care and patient satisfaction with this approach. *The Korean Journal of Internal Medicine*.

[19] Chick A., Wynne A. (2020). Introducing an oral care assessment tool with advanced cleaning products into a high-risk clinical setting. *The British Journal of Nursing*.

[20] Blaschke S. M., Gough K. C., Chua B. H. (2019). Implementation of a multidisciplinary model of care for women with metastatic breast cancer: challenges and lessons learned. *Clinical Breast Cancer*.

[21] Cornelius L. A., Fields R. C., Tarhini A. (2021). Multidisciplinary care of BRAF-mutant stage III melanoma: a physicians perspective review. *The Oncologist*.

[22] Bayliss E. A., Bhardwaja B., Ross C., Beck A., Lanese D. M. (2011). Multidisciplinary team care may slow the rate of decline in renal function. *Clinical Journal of the American Society of Nephrology*.

[23] Dong Q., Zhang Y. (2021). The effect of the prospective information-based nursing quality management model on the improvement of management quality in emergency medicine nursing management. *American Journal of Translational Research*.

[24] Wang Z., Cheng Y., Li J., Hu X. (2021). Effect of integrated medical and nursing intervention model on quality of life and unhealthy emotion of patients with esophageal cancer undergoing radiotherapy. *American Journal of Translational Research*.

[25] Piya M. K., Fletcher T., Myint K. P., Zarora R., Yu D., Simmons D. (2022). The impact of nursing staff education on diabetes inpatient glucose management: a pilot cluster randomised controlled trial. *BMC Endocrine Disorders*.

[26] Fang Q., Li Z. (2019). Effects of hierarchical nursing model on the professional ability and nursing quality of ICU intensive care workers. *Chinese and Foreign Medical Research*.

[27] Zhao R., Lihong L. I. (2019). Evaluation on the application effect of nurse hierarchical nursing management mode in nursing management. China continuing. *Medical Education*.

[28] Chen Y., Yan Z., Hu X., Wei X. (2019). Effects of collaborative nursing mode on the self-management behavior and quality of life in maintenance hemodialysis patients. *Clinical Medicine & Engineering*.

[29] Yang Y., Chen J., Xu D., Wei Y. (2019). The effect of integrative health management model on the nursing care of PICC patients and their quality of life. World latest medicine. *Information*.

[30] Zhang H. T., Wang Y., Room O. (2019). Effect of the optimized management of operating room combined with high quality nursing on improving the quality of nursing in operating room. *Clinical Research and Practice*.

[31] Yuan Y., Oncologynecology D. O. (2019). Analysis on the influence of PDCA combined with ABC nursing management health education for the sleep quality and quality of life of patients with chemotherapy for ovarian cancer. *World Journal of Sleep Medicine*.

[32] Fan X. R. (2019). Analysis of the effect of hierarchical management mode on improving the quality of urological nursing Managemen. *China Health Industry*.

[33] Feng W., Xie H., Ding L., Ruan Y., Zhu Y. (2019). The effect of MDT mode on improving the self-management ability of pregnant women with gestational diabetes mellitus. Chinese. *Nursing Management*.

[34] Zhang Y., Xia M., Liu J. (2019). The effect of synergetic nursing mode on self-management ability of T2DM patients with yin deficiency and fever after discharge from hospital. *Chinese Medicine Modern Distance Education of China*.

[35] Chun Y. E., Center H. (2019). The effects of FOCUS-PDCA procedure combined with supportive psychotherapy on psychological NNquality of life and complications of patients undergoing hemodialysis. *Practical Journal of Clinical Medicine*.

